# Diet impacts on the biological aspects of pink bollworm, *Pectinophora gossypiella* (Lepidoptera: Gelechiidae) under controlled laboratory conditions

**DOI:** 10.1371/journal.pone.0258431

**Published:** 2021-11-11

**Authors:** Arbab Ihsan, Khalid Ali Khan, Muhammad Sagir, Ahmad Nawaz, Sajid Fiaz, Farkhanda Yasmin, Majeeda Rasheed, Habib Ali, Musarrat Shaheen, Samy F. Mahmoud, Samy Sayed, Shafeeq Ur Rahman, Yasir Bilal, Muhammad Ramzan, Talha Nazir, Shumaila Khan, Muhammad Mohsin Waqas, Muhammad Tayyib, Fiaz Hussain, Muhammad Yousaf Ali

**Affiliations:** 1 Integrated Pest Management Laboratory, Department of Entomology, University of Agriculture, Faisalabad, Pakistan; 2 Research Center for Advanced Materials Science (RCAMS), Unit of Bee Research and Honey Production, Biology Department, Faculty of Science, King Khalid University, Abha, Saudi Arabia; 3 Department of Chemical Engineering, Khwaja Fareed University of Engineering and Information Technologies (KFUEIT), Rahim Yar Khan, Punjab, Pakistan; 4 Haripur University, Haripur, Pakistan; 5 Department of Biosciences and Technology, Khawja Fareed University of Engineering and Information Technology, Rahim Yar Khan, Pakistan; 6 Department of life Sciences, Khawja Fareed University of Engineering and Information Technology, Rahim Yar Khan, Pakistan; 7 Department of Agriculture Sciences/Engineering, Khwaja Fareed University of Engineering and Information Technology, Rahim Yar Khan, Pakistan; 8 Cotton Research Institute, Rahim Yar Khan, Pakistan; 9 Department of Biotechnology, College of Science, Taif University, Taif, Saudi Arabia; 10 Department of Science and Technology, University College-Ranyah, Taif University, Taif, Saudi Arabia; 11 Farmland Irrigation Research Institute, Chinese Academy of Agricultural Sciences, Xinxiang, P.R. China; 12 Department of Environmental Sciences and Engineering, Government College University, Faisalabad, Pakistan; 13 Aridzone Research Institute, Bhakkar, Pakistan; 14 Department of Plant Protection, Faculty of Agricultural Sciences, Ghazi University, Punjab, Pakistan; 15 Bahauddin Zakariya University Sub Campus Bahadur-Layyah, Layyah, Punjab, Pakistan; 16 Research & Education Development, Rural Education & Economic Development Society (REEDS), Punjab, Pakistan; Anhui Agricultural University, CHINA

## Abstract

**Background:**

Pink bollworm, *Pectinophora gossypiella* (Lepidoptera: Gelechiidae) is a native pest of Asia and preferably invasion on cotton (*Gossypium hirsutum* L.) crop as a commendatory host plant. Commercially, *G*. *hirsutum* is known as white gold and is an important cash crop all over the globe. Limited studies were published to focus on certain dietary compositions against different cotton pests. Therefore, the present study was undertaken in the laboratory under controlled conditions (temperature: 27 ± 2°C and relative humidity: 60 ± 10%) to determine the impact of three different treatment diets (wheat germ meal, okra, and chickpea) on the biological aspects (lifetime, developmental period) of *P*. *gossypiella*.

**Results:**

Results revealed that the shortest larval time of *P*. *gossypiella* was observed on the okra feed diet while the longest period was recorded on the wheat germ diet. Meanwhile, the pupation delay was noted on the wheat germ diet. The dietary influence was also observed on adult stages of female and male *P*. *gossypiella* (43.00 and 37.50 days respectively) and compared with a standard diet (56.50 and 52.50 days respectively). Furthermore, larval weighed more on the okra and chickpea diet followed by the wheat germ diet, whereas highest pupal weight was observed on the standard diet followed by the chickpea diet and okra diet.

**Conclusion:**

Developmental parameters were significantly variant across all treatment diets, whereas the higher significant difference was reported on the okra diet. Therefore, the existing data of this study offers fruitful interventions for the future as a modified diet for large-scale and rapid mass production of *P*. *gossypiella* larvae.

## Background

Cotton, *Gossypium hirsutum* (L.) also known as white gold and is an important cash crop of Pakistan. Pakistan ranks as the 4^th^ largest producer and 5^th^ largest consumer of cotton in the world. Cotton is cultivated all over the globe with an estimated 32 million hectares for fiber, oil content, fuel, and employment needs [1]. Cotton contributed 0.8% to the gross domestic product (GDP) of Pakistan, whereas, yield decreased to 6% due to unfavorable weather conditions and severe attack of *P*. *gossypiella* that hampered cotton output (Pakistan Economic Survey 2019–20). Genus *Gossypium* belongs to the family Malvaceae recorded as a potential host for *P*. *gossypiella* [2]. Excluding cotton, alternative host plants of *P*. *gossypiella* over the globe can be categorized into 7 families, 24 genera, and 70 species. Among lepidopterans pests (bollworms) of cotton, pink bollworm (Lepidoptera: Gelechiidae) is a native pest of Asia and also prevalent in cotton cultivated areas of the world. It prefers cotton as a host plant to induce injury at its different growth stages [3].

*P*. *gossypiella* lay single white greenish eggs or a bunch of 15 or 20 eggs that change color before hatching [4]. Eggs hatch to neonate larva (2 mm) in 3–4 days with a yellowish and dark brown head, slowly attain a size of second instar (4 mm) having white color then turns to third instar (6 mm) possesses visible pink markings to appear against creamy to ivory background color [5]. Fully grown pink color fourth instar attain a size of 9 mm, feed inside the boll, then exit the boll by making a 2 mm cut and drops to the soil to pupate in case of the short cycle or go to diapause in case of the long cycle when days are short and temperature is falling. Bright brown pupae (7–10 mm long) remains immobile for 7–10 days, then matures into black pupae [6] which emerges into a small inconspicuous greyish moth (12-20mm) with dark spots on wings [5]. The female moth can lay up to 100–200 eggs after 2 days of the pre-oviposition period which can cause severe infestation at the early stage of cotton bolls that cause severe crop loss until quite late in the season. Pink bollworm larval period is 15–20 days and the life cycle is completed in 30–40 days. The principle to control it way is to monitor it at its close season and control the first instar stage that can prevent it from severe crop loss [7].

Many environmental, as well as laboratory-controlled factors [8], affect the developmental period of pink bollworm such as temperature at 29°C shorten incubation period of pink bollworm eggs, whereas coolest temperature [9] and longer exposure of reared larvae to 70°F temperature causes delayed pupation in them [10]. Both pupal period and total life span of pink bollworm vary with the type of food as shorter pupal and egg to emergence period of pink bollworm when fed as larvae on cotton squares compared to feed on cotton bolls [11]. Diet composition also affected the biology of pink bollworm as the higher fat content of the diet resulted in delayed pupation thus increase the incidence of diapause larvae [12–15]. Increased pupal weight increased larval period but reduced pupal weight. However, if the fat content of the diet is lower than the requirements would cause incomplete development of body features and also affect adult emergence [9]. The lower water content of the diet delayed pupation and increased diapause chances [16].

Mass rearing had intense effects on insect performance through first-hand rearing and so has a significant role in integrated pest management [17]. Commercial companies use mass-reared colonies of insects to evaluate pesticide effects, resistance in the host plant, production of replaced products of insect control include viruses, pheromones. The rearing of beneficial insects has great significance for growing industries to increase production and pest control. Many companies use reared insects as intercessors in medicinal products and agriculture [18]. Insect rearing technology involves producing a high number of quality strengthen laboratory insects that benefit entomology for different purposes [19]. As compared to rearing on natural food, rearing on artificial diet optimized to increased insect fitness, lessens the requirement of work effort, space, time, and expenses linked with the growth of host plants and also accessibility of artificial food helps in easier concur of insect growth [20].

The purpose of this study was to determine the impacts of different diet compositions on the developmental, larval and pupal weight of pink bollworms by separately rearing their larvae in reared cups to strictly avoid any contaminations.

## Methods

### Insect collections

For the pink bollworms egg collection, matured cotton bolls were collected from March to May from the cotton fields at The University of Agriculture, Faisalabad (UAF). The cotton bolls that possess diapause larvae (Fig 1) were transferred to glass cages in Pink Bollworm Rearing Laboratory, at the Department of Entomology, UAF under controlled laboratory conditions at 27 ± 2°C temperature and 70 ± 10% relative humidity (RH) that facilitated pupae development to adult emergence. Emerged adults in 1: 1 ratio of male to female was released in oviposition glass chimneys covered with towel tissue paper (white) as an egg lying substrate and provided with vial possessed adult diet (decavitamin drop: 1ml and 10% honey solution) for egg laying purpose. After 3 days of the preoviposition period, collected eggs from the ventral side (possessed grooves) of tissue paper followed shifting to plastic cups for egg hatching (Fig 2).

**Fig 1:** **A-B:** Pink bollworm moth collection cages. **C:** Infested cotton boll due to larval penetration of *P*. *gossypiella*. **D:** Larva feed inside the seed**. E:** Diapause larva under controlled laboratory condition.

**Fig 2:** **A:** Pink bollworm moth collection vial. **B:** Egg laying glass chimney covered with oviposition substrate (groves). **C:** Eggs laid in batches. **D**: Singly egg laid pattern in groves in towel tissue.

### Starter culture

In maintained laboratory conditions, eggs hatched in 2–3 days. Before shifted neonate to rearing cups, noted eggs hatchability percentage because many damaged eggs (attacked by a predator or parasitoid) were not hatched that could further affect larval culture. Plastic cups containing neonate were exposed to torchlight that facilitated their transference to rearing cups (3.8x3.4x3cm) using a camel hair brush (Fig 3). Egg hatchability was checked daily to buildup larval culture for rearing purposes and transferred the hatched larvae to cups possessed diet for mass rearing of pink bollworm adults.

**Fig 3:** **A:** plastic cup possessed many neonates. **B:** Shifting of neonates using camel hair brush. **C:** Rearing cup possessed larvae from starter culture.

### Experimental diets

Three treatment diets including standard diet (the wheat germ as the main ingredient), okra diet, and chickpea symbolized as T1, T2 and T3 were prepared differently according to their suggested formulations. Details of each diet composition are given in Tables 1 and 2. To avoid fungal contamination during diet preparation, firstly sterilized required equipment with 5% ethanol solution (25ml water) followed by autoclave were used. The standard diet prepared based on the technique suggested by [15] is given in Table 1. All ingredients were accurately weighed using electronic balance followed by three fractions (A, B, and C) of ingredients so a well mixed product can be obtained. Fraction A ingredients stirred well in 230 ml of distilled water in a 1000ml of measuring beaker. Then fraction B comprised of decavitamins (0.0l ml) was separately mixed in 10 ml of water in a measuring cylinder to make vitamin solution and then fraction C comprised of agar as a thickening agent was separately well stirred in 500ml of distilled water in a 1000ml of measure beaker followed by boiling it in the oven to make a uniform agar solution. After making fraction solutions, all fractions were blended step by step with the addition of 3.3 ml corn oil and 2 ml honey into a blender mixture followed by pouring of hot mixture into the Petri dishes (150mmx15mm) and allowed to solidify for 10 minutes. The solidified medium was cut with a spatula into small cubes (¼ inches) and placed in 3–4 diet cubes in a transparent plastic cup separately for the rearing of pink bollworm larvae.

**Table 1:** Wheat germ meal artificial diet and its gradients used in this study.

Components of Fraction A	Quantity (g.kg^-1^ or ml. L^-1^)	Components of Fraction B (Decavitamins: 0.01ml)	Quantity (mg.ml^-1^)
Wheat germ meal	34.5	Calcium pentothenate	0.12
Casein	30.0	Niacin	0.06
Sucrose	10.0	Riboflavin	0.03
Brewer’s yeast	5.0	Folic acid	0.03
Alpha-cellulose	1.0	Thiamine	0.015
Potassium sorbate	1.5	Pyridoxine hydrochloride	0.015
Nipalgin	0.5	**Components of Fraction C**	**Quantity (g.kg**^**-1**^ **or ml. L**^**-1**^**)**
Choline chloride	0.06	Agar-agar	20.0
Maize oil	3.3	Distilled Water	500ml
Honey	2.0		
Distilled Water	230		

**Table 2:** Ingredients of chickpea medium along with their quantity.

Components of Fraction A	Quantity (g. ml^-1^)
Chick pea flour	35
Sucrose	15
Distilled Water	200
**Components of Fraction B**	
Agar-agar	19
Distilled Water	200
**Components of Fraction C**	
Dried yeast powder	8.0
Ascorbic acid	1.2
Methyl 4-hydoxy benzoate	1.6
Multivitamin solution	1.0
Streptomycin sulphate	0.2
Bavistin	2.0
Casein	10
Cystiene	0.1
Wesson’s salt	2.5
Sorbic acid	0.5
Cholesterol	0.5

We collected fresh okra fruits (soft and fresh pods) from different fields of UAF then transfer them to pink bollworm rearing laboratory for pink bollworm larval diet. Firstly, we washed okra fruit with distilled water followed by drying then cut 15cm okra with cutter into 2.5 cm okra pieces and placed 5 okra pieces in each transparent plastic cup for larval rearing (Fig 4).

**Fig 4:** Rearing cups possessed okra diet pieces used for larval rearing.

Chickpea diet ingredients and preparation techniques were the same as developed by [21] and given in Table 2. Made three fractions of ingredients, labelled as A, B and C then mixed fraction A’s ingredients in 200ml of distilled water, warmed to 60°C with continuous stirred followed by cooling then added dissolved solution into a blender and mixed thoroughly. Then fraction B comprised of agar was boiled in 200 ml of distilled water in an oven followed by continued stirring until beading consistency was obtained, then blended dissolved viscous agar into fraction A. Finally, fraction C ingredients were added into fraction A mixture with continuous blending until a homogenous mixture was obtained. The prepared diet was poured into Petri dishes and diet cubes (2cm × 0.2cm × 0.5cm) were placed in rearing containers for larval rearing.

### Experimental layout

The experiment was set up in a completely randomized design (CRD) comprised of three treatment diets including standard, okra, and chickpea diets and each treatment was replicated 10 times while possessed two larvae per replication.

### Population rearing

After obtaining a successful culture of the neonate, there was a need to shift them on prepared diets for successful rearing. For rearing purposes, small-sized plastic cups with lids were used as reared containers to prevent larval escape, predator entry, diet contamination, and dehydration. Marked transparent plastic cups replicated 10 times for each treatment diet and using camel’s hair brush released freshly emerged neonates onto diet cubes at 2 larvae/cup and reared until pupation. For successful larval development, larvae shifted onto a fresh diet (Fig 5) for every third day while daily observed larval stage and increased diet according to the larval stage. The fourth stage larvae were sexed, weighed, and counted separately for adult pairing. Upon pupation, the pupae were weighed and transferred dark brown pupa in wide-mouthed specimen jars labelled as male and female for separate adult emergence and collection. After the pupation, the emerged adults were released in pairs into oviposition glass chimneys for mating and egg-laying purpose. Wide-mouthed round glass chimneys were used to prevent excessive flight activity, crowding of adults, preserve scales and facilitate mating among adults.

**Fig 5:** 1: Neonate larva shifted on diet **2:** Second instar larva feed on prepared diet **3:** Third instar **4:** Fully grown fourth instar ready to pre-pupate **5:** Male and female dark brown pupae **6:** Emerged pink bollworm adult.

### Statistical analyses

Observations on biological parameters including incubation, larval, pupal, larval period and pupal weight, adult longevity and mean generation time were recorded for each larval diet and subjected to appropriate statistical analysis using statistical 8.1 software.

## Results

Growth and development records of pink bollworm reared on three treatment diets are given in Table 3. Analysis of variance records indicates the instar duration of each larval stage significantly differed across three treatment diets. Instar period of newly hatched larvae was observed to be the shortest on the chickpea diet followed by the okra diet as compared to the standard diet, while [22] reported 2.34 ± 0.48 days for the first instar period on chickpea diet agreed with the present findings on chickpea diet. According to statistical analysis (Fig 6), the first instar period (2.4b) was noted to be significantly different on the chickpea diet as compared with the non-significant differences in the second instar period between standard and okra diet (3.6a and 3.4a).

**Fig 6:** Larval instar’s duration (mean ±SE) of *P*. *gossypiella* on wheat germ, okra and chickpea diet. The means followed by each instar’s bar gram by same letters are not significantly different at p>0.05 by Tukey’s HSD test.

**Table 3:** Growth and development of *Pectinophora gossypiella* reared on various treatment diets.

Diet	Biological Parameters (Days)									
	1st Instar	2nd Instar	3^rd^ Instar	4^rth^ Male Instar	4^rth^ Female Instar	Male Larval period	Female Larval period	Pupal period	Male life Cycle period	Female life Cycle period
Wheat germ meal	3.6a	4.7a	4.9a	6.2a	8.4a	19.4a	21.6a	8.6a	52.5a	21.0a
Okra	3.4a	3.5b	3.5b	3.7b	4.2b	14.0c	14.5b	7.7ab	39.8b	18.5a
Chickpea	2.4b	4.3ab	4.6a	6.2a	8.3a	17.5b	19.6a	7.3b	37.5b	12.1b
HSD value	0.5727	0.9710	0.7929	0.7784	0.7424	1.7457	2.1053	1.1414	3.7493	2.7614
F-Value	15.5**	4.87**	10.6**	42.3**	128**	30.3**	37.2**	4.19**	57.1**	29.4**

** Highly significance difference at 1% probability level; *Significance difference at 5% probability level; NS: no significant difference.

Means within a column shared by same letters are not significantly different at p>0.05 fallowed by Tukey’s test.

The shortest second instar period was noted on the okra diet followed by larvae reared on chickpea diet as compared to the longest period recorded on wheat germ diet while the [15] findings (4.31 ± 0.76 days) slightly deviated from our results recorded on chickpea diet. According to statistical analysis, a significantly higher (4.7a), second instar period was recorded on the standard diet which was significantly different from the okra diet while there was no significant difference in the second instar period between okra (3.5b) and chickpea diet (3.5ab) or between the standard and the chickpea diet. The shortest third instar duration was observed on the okra diet followed by the chickpea diet as compared to the longest period noted on the wheat germ diet while the instar period on the okra diet was in agreement with the [22] results on chickpea diet. The statistical analysis described the third instar duration of *P*. *gossypiella* moth significantly higher (4.9a) on the standard diet but the instar period significantly differed (3.5b) when larvae reared on okra diet compared to those fed on the standard diet and chickpea diet (4.6a) that showed non-significant differences.

The third instar turned to dark pink color, the fourth instar distinct as male and female while both sexes showed different development duration depends on the type of diet on which both reared separately. The shortest period of male fourth instar was observed on okra diet followed by wheat germ diet and longest instar period was noted on chickpea diet which was in synchronism with [22] observations reported for male instar duration of 6.40 ± 0.52 days. Statistically analyzed, the fourth instar period of male larvae was significantly higher and did not significantly differ when fed on standard and chickpea diet (6.2a on both) as compared to okra diet (3.7b) on which significantly differed instar period was observed.

The observed shortest period of female fourth instar on okra diet followed by chickpea diet and longest instar period was noted on wheat germ diet while chickpea findings were in contrast with the [22] findings reported 5.60 ± 0.68 days female instar period on chickpea diet. Statistically analyzed, female fourth instar period was significantly higher on wheat germ diet (8.4a) and non-significantly differed from chickpea diet (8.3a) while significantly differed on okra diet (4.2b)

After the mean instar period was completed, the recorded total larval period as male and female were reared separate treatment diets. The shortest male and female larval was observed on okra diet followed by chickpea diet as compared to longest larval period on wheat germ diet while male larval period on chickpea diet was in line (Fig 7) with [22] findings (17.5 ± 1.95 days) and female larval period was in contrast with the [22] findings (8.15 ± 2.18 days). In present results, larval period recorded on chickpea diet was in conformation with [5] results recorded total larval period range from 18.26–18.96 days on seed powder of cotton cultivars and also in accord with the [23]) findings on hornworm diet. Okra diet findings were in contrast with the [24, 25] who reported the shortest instar period of 21.34 ± 2.61 days on two-phase diets (cottonseed flour and okra).

**Fig 7:** Larval period (mean ±SE) of male and female *P*. *gossypiella* on wheat germ, okra and chickpea diet. The means followed by bar gram by same letters are not significantly different at p>0.05 by Tukey’s HSD test.

Present findings of the larval period on three different diets were in contrast with the earlier studies of [26] reported 11.33±0.64 days; [27] recorded 9 to14 days in the hotter region; Shah *et al*., 2013 noted 9 days at 35 ± 1°C and 13 days at 27 ± 1°C as well as [21] who found it to be 25.10 ± 0.994 days when reared on artificial medium. Larval period reported by [28, 29] was in agreement with the present findings. Statistical analyses indicate that the adult larval period differed highly significantly (P<0.01) when reared on selected larval diets. The present findings of the larval period were in contrast with earlier studies of [30] results reported the non-significant effect of cotton cultivars on pink bollworm larval period; [25] observed non-significant larval period difference across southern pink bollworm diet premix and cottonseed flour + Chickpea flour + okra diet but significant larval period difference noted by [25] on cottonseed flour, cottonseed flour + chickpea flour, cottonseed flour plus okra and southland multi-species diet premix that conformed with present findings.

Male larval period significantly differed across three treatment diets as lengthy male larval period observed when reared on the standard diet (19.4a) followed by reared on chickpea diet (17.5b) as compared to reared on the okra diet (14.0c). Female larval period significantly higher (21.6a) when larvae reared on the standard diet which differed non-significantly from larval period observed on the chickpea diet (19.6a) while significantly differed larval period (14.b) was observed on the okra diet. After the completion of larval development, the fourth instar larva of pink bollworm went to diapause state as it stopped feeding and moved slow, as a resulted in its body stretched and shield-like covering formed on body identified as the pre-pupal stage. The prepupal stage short that turns into the resting stage called the pupal stage in which developmental structures formed. The pupal period varied depending on the type of diet larvae reared.

As recorded from Table 4 the longest pupal duration recorded on the standard diet which was in agreement with [31] results reported 8 days pupal period at 35 ± 1°C and also slightly in accord with [32], findings reported 8.8 days on wheat germ diet. Pupal period recorded on standard diet was also in agreement with [28] findings on the cotton square, wheat germ, and modified wheat germ diet and in accord with the Bell and [33] findings on hornworm diet. Recorded shortest pupal period of larvae reared on chickpea diet which was in accordance with the [22] findings on chickpea die and more or less in agreement with [26] who found the pupal period consisting of 7.42 ± 0.20 days.

**Table 4:** Mean comparison of larval and pupal weights of pink bollworm reared on three treatment diets.

Diet	Larval weight	Pupal weight
	(mg)	(mg)
Wheat germ meal	17.6a	21.2a
Okra	19.6a	16.4b
Chickpea diet	19.4a	17.4b
HSD value	2.2700	1.9042
F-value	3.37^NS^	25.3**

**Significance difference at 1% probability level; *Significance difference at 5% probability level; NS: no significant difference.

Means within a column shared by same letters are not significantly different at p>0.05 fallowed by Tukey’s test.

## Discussion

In contrast to present findings, Kandi (2016) recorded pupal period as 16.7 days at 25°C, [34] found 3.5 days pupal delayed at the varied temperature of 18 to 35°C, [25] reported the shortest pupal period of 7.96 ± 1.37 days when larvae reared on two-phase diets (cottonseed flour and okra), [21] recorded pupal period of 7.9± 0.88 days when reared on artificial medium, [30] noted pupal period ranging from 5.76–6.48 days when artificially reared larva on seed powder of cotton cultivars. According to statistical analysis, the pupal period of *P*. *gossypiella* differed significantly (P<0.05) across treatment diets. Similar to present results, the pupal period reported by [30] significantly differed on some cotton cultivars (G-27, Pusa 1752 and Gh-BHV-824) and the pupal period reported by [25] significantly differed on cottonseed + chickpea flour, cottonseed flour, southland multispecies diet premix.

Pupal period significantly higher (8.6a) and significantly differed when larvae reared on wheat germ diet than those reared on okra (7.7ab) and chickpea diet (7.3b) which show a non-significant difference in the pupal period. Similar to the present results, [25] found a significantly lengthen pupal period (8.78 ± 1.70c) on cottonseed flour + chickpea flour diet as compared to the non-significant shorter pupal period on other combinations of diets. The total life cycle period of pink bollworms depends on the type of diet on which larvae reared. According to the table, the longest life cycle period from egg to adult of female and male was recorded on the standard diet but only female total life span was in agreement while male life cycle period deviated from [22] findings who reported 56.30 ± 9.84 and 38.40 ± 4.48 days on chickpea diet. The developmental period of females and males on the okra die was in confirmation with [35] conclusions who reported mean generation time from egg to egg as 37.8 ± 3.8 days and is in agreement with [36, 37] findings. The total life span of female and male moth reared on chickpea diet was in accordance with reported results who noted female developmental period of 21 to 43 days. Present findings were contrary to earlier studies of [38] who described the total life cycle period of 25–30 days and [31] reported 30–32 days at 35 ± 1° C.

Statistical analysis (Fig 8) indicates that male and female life cycle periods differ highly significantly (P<0.01) on three treatment diets. Male life cycle period significantly higher (52.5a) when larvae reared on a standard diet and significantly differed from okra diet (39.8b) that non-significantly differed from chickpea diet (37.5b). Female life cycle period significantly higher (56.5a) on a standard diet and significantly differed from total life span observed on chickpea diet (43.9b) that non-significantly differed from okra diet (43.6b). Data from Table 3, larval weight observed highest on okra and chickpea diet followed by wheat germ diet. Pupal weight is an indicator of food conversion efficiency during larval stages, which was observed the highest on standard diet followed by chickpea diet and okra diet. Present findings on standard diet were in conformation with [39] results on processed cottonseed meal diets while the larval and pupal weight on okra and chickpea diet was in conformation with [21] findings who reported 21.40 ± 3.63 and 18.00 ± 2.73 mg weight. According to statistical analysis (Fig 9), larval weight was not different significantly (P>0.05) when reared on three treatment diets whereas significantly higher larval weight was observed when larvae fed on okra diet(19.6a) as compared to chickpea (19.4a) and standard diet (17.6a). While pupal weight differed significantly (P<0.05) across treatment diets which was inconsistent with the results recorded by [25] as pupal weight significantly differed on cottonseed flour + Okra, cottonseed flour + chickpea flour, and southland pink bollworm diet premix. Pupal weight was observed significantly higher (21.2a) and significantly differ on standard diet as compared to chickpea (17.4b) and okra diet (16.4b) that showed non-significant differences. Present results are in line with the [25] who recorded significantly highest pupal weight (21.78 ± 4.09a) on cotton.

**Fig 8:** Total life span (mean ±SE) of male and female *P*. *gossypiella* on wheat germ, okra and chickpea diet. The means represent by bar gram by same letters are not significantly different at p>0.05 by Tukey’s HSD test.

**Fig 9:** Larval and pupal weight (mean ±SE) of *P*. *gossypiella* on wheat germ, okra and chickpea diet. The means followed by bar gram by same letters are not significantly different at p>0.05 by Tukey’s HSD test.

## Conclusion

The present study facilitates to develop an artificial diet for *P*. *gossypiella* prepared from locally available ingredients and a simple adaptable methodology by different researchers. Okra diet is useful for large-scale mass production of *P*. *gossypiella* due to rare contamination and easy handling whereas, in the case of other diets, contamination chances are high due to poor laboratory tools and mite infestation.

## Abbreviations

GDP: gross domestic product
RH: relative humidity
CRD: completely randomized design
